The article "Evaluation of the Reliability and Quality of YouTube Video Content about Perianal Fistulas" was published in 2022. Journal: Biomed Res Int.

# Evaluation of the Reliability and Quality of YouTube Video Content about Perianal Fistulas

**DOI:** 10.1155/2022/2955273

**Published:** 2022-11-16

**Authors:** Ersan Eroglu, Ediz Altinli

**Affiliations:** Department of General Surgery, Memorial Bahcelievler Hospital, Istanbul, Turkey

## Abstract

**Objective:**

Perianal fistulas of the perianal soft tissues are an important cause of morbidity and a significant portion of colorectal surgery. To our knowledge, there is no study evaluating YouTube videos pertaining perianal fistulas. In this study, we aimed to evaluate YouTube video contents on this topic.

**Methods:**

Whether the videos contained real images, animations or presentations, video duration, number of views, comments and likes, uploading date, and daily view were recorded. Reliability of the videos was assessed using the Quality Criteria for Consumer Health Information (DISCERN) scale and quality of the videos using the Global Quality Score (GQS).

**Results:**

A total of 100 YouTube videos regarding perianal fistulas were included in the study. Sixty-four (64%) videos were uploaded by healthcare professionals and 36 (36%) videos by nonprofessionals. The mean video length was calculated as 6.70 ± 8.00 minutes for all videos. The mean DISCERN score of all videos was found as 3.92 ± 0.81 and the mean GQS score as 3.97 ± 0.83. According to the DISCERN score, most videos included (94%) were of good quality. There was an excellent agreement between the two surgeons in terms of the DISCERN and GQS scores.

**Conclusion:**

Most of the videos included in the study were uploaded by health-care professionals. On the other hand, the majority of the videos contained surgical management of perianal fistulas as it is the definitive treatment. Healthcare related content should be audited and filtered by YouTube with new and effective policies.

## 1. Introduction

Perianal fistulas of the perianal soft tissues are an important cause of morbidity and a significant portion of colorectal surgery (1). Perianal fistula is a common disease, notorious for recurrence if left untreated (2). These fistulas are abnormal connections between two surface lined with epithelium, usually the anal canal mucosa and the perianal skin. It is a rare disease, affecting approximately 0.01% of the general population (3). Perianal fistula frequently occurs in patients with Crohn's disease (4). Treatment of perianal fistulas has changed over years from primary surgical management to multidisciplinary management (5). People with some diseases including perianal fistula often search other sources of information related to their health problem before seeking medical help due to hesitancy, fear of surgery, and searching for alternative treatments.

The article "Evaluation of the Reliability and Quality of YouTube Video Content about Perianal Fistulas" was published in 2022. Journal: Biomed Res Int.

In today's digital world, the internet and especially social media has become an indispensable part of daily life. The Internet has become a popular source of health related information (6). Previous studies have reported that 80% of Internet users access health related information online (7). The Internet is becoming more preferable by patients due to its low cost, 24 h use, anonymous accessibility, and updated data (8).

YouTube is the most commonly used video sharing platform and the second most popular website in the world following Google search (9). Every minute more than 500 h of video content are uploaded to YouTube, and people watch over a billion hours of video (10). YouTube has extended its limit beyond text-based information and became a potential source for spreading medical information through uploaded videos (11).

However there are concerns about the reliability and quality of online health related information. Eighty-six percent of health seekers are concerned about the reliability of information available on the internet, and 44% believe that only part of this information is accurate (12). In a recent study, it was found that more than 25% of the most viewed YouTube videos pertaining COVID-19 contained misleading information that reached millions of people worldwide (13). Although YouTube provides video contents to its consumers free, there is no control mechanism for accuracy and quality of videos. Therefore, YouTube members can upload videos on topics they want, and low quality or nonaccurate information can spread to the society.

Therefore, the number of studies investigating the reliability and quality of YouTube video contents related to various fields of medicine is increasing (14–16). To our knowledge, there is no study evaluating YouTube videos pertaining perianal fistulas. In this study, we aimed to evaluate YouTube video contents on this topic.

## 2. Material and Methods

Ethic committee approval for this study was not obtained, because the study did not include human or animal subjects, and YouTube videos were accessible to anyone, consistently with previous studies (17).

This study was performed by two experienced general surgeons (10-year and 15-year experienced) as a reliability and quality analysis of YouTube videos pertaining perianal fistulas at 05-07/07/2022. Searching terms were determined by consensus of the two surgeons as “perianal fistula” and “perianal fistula treatment”. From filter options of YouTube, the videos were sorted by “relevance” which is the default searching option. Studies have reported that the users mostly review videos on the first three pages of the results (8, 18). After excluding non-English videos, duplicate videos, and those including advertisements, we included the first 100 videos in the analysis. The links of these videos were entered to the Microsoft Excel software and analyzed by the two observers at the same time interval, but in separate places to avoid potential bias between them. Flowchart of the inclusion is seen in Figure 1.

The article "Evaluation of the Reliability and Quality of YouTube Video Content about Perianal Fistulas" was published in 2022. Journal: Biomed Res Int.

### 2.1. Data Collection

Whether the videos contained real images, animations or presentations, video duration, number of views, comments and likes (dislike option was removed by YouTube), uploading date, and daily view were recorded. Daily view was calculated by the formula, (reviewing date − uploading date/total views). Video source was categorized as physician, technician, health channel, patient, and lay person. Physicians and technicians were considered as healthcare professionals and the others as lay persons.

### 2.2. Evaluation of the Videos

Reliability of the videos was assessed using the DISCERN scale and quality of the videos using the Global Quality Score (GQS). These two measurement tools have been widely used in the previous studies (14–16). In addition, the videos included in the analysis were evaluated in terms of usefulness by the consensus of the two researchers as useful and misleading. In line with the previous studies (19, 20), the videos were considered useful if they contained scientifically accurate information about the disease examined or misleading if they contained scientifically unproven information.

### 2.3. DISCERN Scale

DISCERN is a scoring measurement tool for assessment of the reliability of consumers' health information on treatment options. In this study, we used the modified DISCERN tool, which was created for the first time by Charnock et al. and shortened by Singh et al. (11, 21). The scale consists of 5 questions evaluated with a 5-Likert scale between 0 and 5. Higher scores represent greater reliability. Reliability of a video content is considered good for a DISCERN score > 3 points, moderate for a DISCERN score of 3 points and poor for a DISCERN score < 3 points (16).

### 2.4. Global Quality Score (GQS)

GQS scale was developed for the first time by Bernard et al. in order to measure the quality of a video content based on the usefulness of the information offered in the video (22). This scale consists of 5 questions that inquiries quality, flow and easy to use information given in the video with a 5-Likert scale. Higher scores represent greater quality.

The videos included in the analysis were scored independently by the two surgeons. The Kappa coefficient was used for the determination of interobserver agreement.

The article "Evaluation of the Reliability and Quality of YouTube Video Content about Perianal Fistulas" was published in 2022. Journal: Biomed Res Int.

### 2.5. Statistical Analysis

Statistical analysis was performed using the SPSS version 25.0 (SPSS, Statistical Package for Social Sciences, IBM Inc., Armonk, NY, USA) statistical software. Normal distribution of the variables was tested using the Kolmogorov-Smirnov method. The variables were found to be nonnormally distributed. The comparison of the continuous variables between the two groups was made with Mann–Whitney *U* test, while the categorical variables were compared with Chi-Square test. The DISCERN and GQS scores according to video sources were compared using the Kruskal–Wallis test. The continuous variables are expressed as mean ± standard deviation and categorical variables as frequency (*n*, %). Cronbach's alpha coefficients were used to calculate the agreement between the two researchers. *p* < 0.05 values were considered statistically significant.

## 3. Results

A total of 100 YouTube videos regarding perianal fistulas were included in the study. The total view count of all videos was 15,005,136, and the total duration was 11.17 hours. The most common video content was treatment followed by general information and imaging (Figure 2).

Types of images were divided into three groups as real image, animation, and presentation. Accordingly, 82 (82%) videos contained real images; 12 (12%) videos contained presentations, and 6 (6%) videos contained animation.

When qualification of the uploaders was examined, medical doctors uploaded 61 videos, health channels 15 (15%) videos, technicians 3 (3%) videos, patients 4 (4%) videos, and others 17 videos. Therefore, 64 (64%) videos were uploaded by healthcare professionals and 36 (36%) videos by nonprofessionals.

The mean video length was calculated as 6.70 ± 8.00 minutes for all videos. The mean video length was found as 6.74 ± 8.03 in the videos uploaded by professionals and 6.74 ± 8.03 in the videos uploaded by nonprofessionals. There was no statistically significant difference between the professionals and nonprofessionals in terms of the video length (*p* > 0.05). The oldest video was uploaded on October 11, 2011, and the newest video on November 22, 2021. The mean duration since the upload was 1330.50 ± 865.02 days. The mean daily view count was calculated as 104 ± 139. The mean daily view count was found as 104 ± 140 in the professional and 103 ± 139 in the nonprofessional group (*p* > 0.05). The mean number of daily views, comments, and like counts of the videos are given in Table 1.

The videos included in this study were evaluated by the two surgeons subjectively in terms of usefulness. In case of a disagreement, the opinion of a third surgeon was received, and the decision was made on consensus. According to this evaluation, most videos (77%) regarding perianal fistulas were useful, while the others were misleading (23%). This evaluation was made independently from the DISCERN and GQS scoring and regardless of the uploaders.

The article "Evaluation of the Reliability and Quality of YouTube Video Content about Perianal Fistulas" was published in 2022. Journal: Biomed Res Int.

Reliability of the videos was evaluated with DISCERN and quality of the videos with GQS scales. The mean DISCERN score of all videos was found as 3.92 ± 0.81 and the mean GQS score as 3.97 ± 0.83. Distribution of the DISCERN and GQS scores according to the uploaders is presented in Figure 3. Distribution of the DISCERN and GQS scores according to the video content is shown in Figure 4.

Table 2 shows the comparison of DISCERN and GQS scales between professionals and nonprofessionals. According to the DISCERN score, most videos included (94%) were of good quality.

The agreement between the two surgeons was evaluated with Cronbach's *α* coefficient. There was an excellent agreement between the two surgeons in terms of the DISCERN and GQS scores (Table 3).

## 4. Discussion

People with some diseases including perianal fistulas often hesitate to see a doctor to seek a solution for their disease and discomfort. Although rare, perianal fistulas is a painful condition that causes discomfort and impaired quality of life. Within this context, YouTube has an advantage to offer health related information for free in almost all fields of medicine. However, since there is no control mechanism, anyone including lay persons can load any information about health topics that can spread to millions of people. This has prompted researchers to investigate accuracy, quality, and reliability of information in YouTube video contents. The first study on YouTube videos was conducted by Keelan et al. and evaluated the quality of videos related to immunization (23). Since that time, many investigators analyzed YouTube videos associated with various diseases (24–26).

In the present study, we investigated the reliability and quality of YouTube videos pertaining perianal fistulas. In our study, videos included in the analysis contained real images by 82% followed by presentations (12%) and animations (6%). Similarly, in a study by Toprak and Tokat, investigating YouTube videos on nocturnal enuresis, 85.2% of the videos contained real images, and 14.8% contained animation (8). Looking to the DISCERN and GQS scores of the real or animated videos, no significant difference was found between them (*p* > 0.05). In another study by Krakowiak et al., the rate of animated videos was reported as 26% with higher DISCERN scores (27). In a study by Gokcen et al., no difference in quality was found between the real and animated videos (28). This difference might be attributed to differences between of topics of interest. Since definitive treatment in perianal fistulas is surgical treatment, videos contained both real images and animations included surgical treatment, and the scores were similar between them.

The article "Evaluation of the Reliability and Quality of YouTube Video Content about Perianal Fistulas" was published in 2022. Journal: Biomed Res Int.

Length of health related videos on YouTube differs widely among the studies depending on the topic of research. In our study, the mean length of all videos was 6.70 ± 8.00 minutes. In the study by Toprak et al. this duration was found as 3.61 minutes. In another study by Duran and Kizilkan on quality analysis of testicular cancer videos on YouTube, the mean video length was reported as 8.86 minutes (29). In another study by Zengin and Onder, the mean video length was found as 4.21 minutes (30). The mean video length found in our study was within the range reported by the other studies.

In our study, 61 videos were uploaded directly by physicians, 17 by lay persons, 15 by health channels, 4 by patients, and 3 by technicians. When examining the contents of the videos, we considered the videos uploaded by physicians and technicians as professional and the others nonprofessional videos. Accordingly, 64% were uploaded by professionals and 36 by nonprofessionals. The mean daily view count was found as 104 ± 140 in the professional and 103 ± 139 in the nonprofessional group (*p* > 0.05).

In a study by Chang and Park, investigating YouTube videos regarding exercises and compensated maneuvers for dysphagia, 20 videos were uploaded by universities/professional organizations, 14 videos by therapists, 10 videos by health related websites, and 4 videos by physicians (31). In the study by Toprak and Tokat, 26 videos were uploaded by physicians, 12 videos by health-related websites, 7 videos by TV programs, and 4 videos by patients (8). As seen, qualification of the uploaders varies according to the research topic. However, the examined videos were largely uploaded by professionals as in the present study. Previous studies also reported that the most common uploaders of the videos were physicians (32).

Interestingly, like and comment counts were significantly higher in the videos uploaded by nonprofessionals. This may be attributed to the fact that physician's narration during the video may contain medical terminology that everyone cannot understand exactly. On the other hand, Toprak and Tokat found that the number of likes and comments were not indicators of video quality (8).

In the current study, we evaluated DISCERN and GCS scores according to uploaders and video contents. Accordingly, physicians had the highest DISCERN and GCS scores followed by health channels, while patients had the lowest scores. However, even in some videos directly uploaded by physicians, there was no narration or any explanation except for the real images during surgery. Considering video contents, education had the highest scores followed by treatment and general information. Almost all treatment-related videos contained surgical treatment for perianal fistulas with real images and narration, which is the definitive solution for perianal fistulas. In the literature, the highest scores for DISCERN and GQS were considered to indicate the highest reliability and quality, which was also the case in our study (8, 14–16, 29).

The article "Evaluation of the Reliability and Quality of YouTube Video Content about Perianal Fistulas" was published in 2022. Journal: Biomed Res Int.

### 4.1. Study Limitations

One of the major limitations was taking snapshots of information, but YouTube has a dynamic structure, and new contents are updated constantly. Another limitation was that we only analyzed English-language videos. However, English is accepted as the prevailing language for access to online information. Finally, the video assessment process was subjective, although interrater agreement was excellent.

## 5. Conclusion

Most of the videos included in the study were uploaded by health-care professionals. And most of them were evaluated as useful. However, the mean reliability and quality scores were low even for some videos uploaded by physicians such as videos with music alone without any speech or explanation. On the other hand, the majority of the videos contained surgical management of perianal fistulas as it is the definitive treatment. Healthcare related content should be audited and filtered by YouTube with new and effective policies.

## Figures and Tables

**Figure 1:** Flow chart of the video inclusion.

**Figure 2:** Distribution of videos regarding perianal fistulas by video content.

**Figure 3:** DISCERN and GQS scores by uploaders.

**Figure 4:** DISCERN and GQS scores by video contents.

**Table 1:** Basic characteristics of the videos reviewed.

Feature	Daily views	Comments	Likes
	Mean ± SD	Mean ± SD	Mean ± SD
*Image type*			
Real (*n* = 82)	96.15 ± 127.95	95.26 ± 265.63	716.85 ± 1997.79
Presentation (*n* = 12)	59.74 ± 117.24	40.75 ± 46.55	679.30 ± 959.04
Animation (*n* = 6)	250.32 ± 221.42	53.60 ± 68.54	1278.17 ± 1385.72
*Uploaders*			
Medical doctors (*n* = 61)	103.10 ± 133.96	85.15 ± 122.70	607.69 ± 785.15
Technicians (*n* = 3)	64.37 ± 97.34	20.33 ± 32.65	358.67 ± 555.41
Health channels (*n* = 15)	164.24 ± 184.13	37.31 ± 49.14	965.57 ± 1193.2
Patients (*n* = 4)	13.73 ± 8.72	115.50 ± 154.86	122.00 ± 124.45
Others (*n* = 17)	71.80 ± 118.61	145.24 ± 527.47	1193.65 ± 4079.74
*Professionals vs. lay persons*			
Professionals (*n* = 64)	101.10 ± 131.94	81.79 ± 120.45	595.44 ± 773.87
Nonprofessionals (*n* = 36)	102.94 ± 150.54	99.53 ± 384.83	1031.94 ± 2994.76
*Video content*			
General information (*n* = 29)	82.93 ± 106.92	45.73 ± 57.35	553.93 ± 760.84
Treatment (*n* = 52)	122.33 ± 152.30	72.31 ± 110.31	633.10 ± 851.62
Imaging (*n* = 8)	31.67 ± 221.90	11.33 ± 270.77	202.29 ± 355.74
Examination (*n* = 1)	226	139	2100
Alternative medicine (*n* = 2)	352.12 ± 350.22	1101.00 ± 1538.66	8551.50 ± 11947.98
Education (*n* = 3)	29.88 ± 23.76	13.33 ± 19.66	56.33 ± 19.86
Patient experience (*n* = 4)	13.73 ± 8.72	115.50 ± 154.86	122.00 ± 124.45

The article "Evaluation of the Reliability and Quality of YouTube Video Content about Perianal Fistulas" was published in 2022. Journal: Biomed Res Int.

**Table 2:** DISCERN and GQS of professionals and nonprofessionals.

	*n* (%)	DISCERN	GQS	*p* value
		Mean ± SD	Mean ± SD	
*Uploaders*				
Professionals	64 (64)	3.91 ± 0.82	3.97 ± 0.84	<0.05
Nonprofessionals	36 (36)	3.85 ± 0.80	3.88 ± 0.84	

**Table 3:** Agreement between the two surgeons.

	Mean ± SD	*p*	*r*	Cronbach's *α*
DISCERN 1	3.89 ± 0.85	*p* < 0.01	0.888	0.89
DISCERN 2	3.94 ± 0.90			
GQS 1	3.95 ± 0.86	*p* < 0.01	0.895	0.91
GQS 2	3.99 ± 0.89			

## Data Availability

Data used in this study can be provided on reasonable request.
